The article "Sanhua Decoction, a Classic Herbal Prescription, Exerts Neuroprotection Through Regulating Phosphorylated Tau Level and Promoting Adult Endogenous Neurogenesis After Cerebral Ischemia/Reperfusion Injury" was retracted in 2024. Reasons: unreliable data; unreliable results or conclusions; concerns about the images.

# Sanhua Decoction, a Classic Herbal Prescription, Exerts Neuroprotection Through Regulating Phosphorylated Tau Level and Promoting Adult Endogenous Neurogenesis After Cerebral Ischemia/Reperfusion Injury

**DOI:** 10.3389/fphys.2020.00057

**Published:** 2020-02-11

**Authors:** Deng-Lei Fu, Ji-Huang Li, Yi-Hua Shi, Xi-Le Zhang, Yan Lin, Guo-Qing Zheng

**Affiliations:** Department of Neurology, The Second Affiliated Hospital and Yuying Children’s Hospital of Wenzhou Medical University, Wenzhou, China

**Keywords:** traditional Chinese medicine, ischemic stroke, endogenous neurogenesis, tau phosphorylation, neurological function recovery

## Abstract

**Background:** Ischemia stroke is the leading cause of death and long-term disability. Sanhua Decoction (SHD), a classic Chinese herbal prescription, has been used for ischemic stroke for about thousands of years. Here, we aim to investigate the neuroprotective effects of SHD on cerebral ischemia/reperfusion (CIR) injury rat models.

**Methods:** The male Sprague-Dawley rats (body weight, 250–280 g; age, 7–8 weeks) were randomly divided into sham group, CIR group, and SHD group and were further divided into subgroups according to different time points at 6 h, 1, 3, 7, 14, 21, and 28 d, respectively. The SHD group received intragastric administration of SHD at 10 g kg^−1^ d^−1^. The focal CIR models were induced by middle cerebral artery occlusion according to Longa’s method, while sham group had the same operation without suture insertion. Neurological deficit score (NDS) was evaluated using the Longa’s scale. BrdU, doublecortin (DCX), and glial fibrillary acidic protein (GFAP) were used to label proliferation, migration, and differentiation of nerve cells before being observed by immunofluorescence. The expression of reelin, total tau (t-tau), and phosphorylated tau (p-tau) were evaluated by western blot and RT-qPCR.

**Results:** SHD can significantly improve NDS at 1, 3, 7, and 14 d (*p* < 0.05), increase the number of BrdU positive and BrdU/DCX positive cells in subventricular zone at 3, 7, and 14 d (*p* < 0.05), upregulate BrdU/GFAP positive cells in the ischemic penumbra at 28 d after CIR (*p* < 0.05), and reduce p-tau level at 1, 3, 7, and 14 d (*p* < 0.05). There was no significant difference on reelin and t-tau level between three groups at each time points after CIR.

**Conclusions:** SHD exerts neuroprotection probably by regulating p-tau level and promoting the proliferation, migration, and differentiation of endogenous neural stem cells, accompanying with neurobehavioral recovery.

## Introduction

Ischemic stroke is caused by occlusion of cerebral vessels, which ultimately results in irreversible brain damage. According to recent global epidemiological researches, ischemic stroke has been a leading cause of death and long-term disability, causing a huge burden on both patients and society (Meyers et al., 2011; Naghavi et al., 2017; Venketasubramanian et al., 2017; Pandian et al., 2018). Circulation reconstruction is important especially for salvage of ischemic penumbra, which contributes to minimize neurological deficits (Belayev et al., 2018). Effective therapy is still limited. Intravenous recombinant tissue-type plasminogen activator is a recommended pharmacological effective therapy (National Institute of Neurological Disorders and Stroke rt-PA Stroke Study Group, 1995; Powers et al., 2018); however, there is though it not only has strict therapeutic time window but also may cause serious complications such as hemorrhage (Sandercock et al., 2012; Berge et al., 2016; Demaerschalk et al., 2016). Moreover, most patients remain neurological deficits, even if they have received effective intravenous thrombolytic therapy (Grabowska-Fudala et al., 2018). Another approved effective treatment is thrombectomy within 24 h (Nogueira et al., 2018); but only a few right patients in the right place within the right time frame can be implemented the mechanical thrombectomy because a comprehensive stroke unit and a group of qualified neurointerventionalists are required for performing the surgery.

Neural stem cells (NSCs) can proliferate and divide into neural precursor cells (NPCs), migrate, differentiate into mature neurons, and then form synaptic connections with surrounding cells. In the central nervous system (CNS), NPCs have been found mainly located in the subventricular zone (SVZ) and the subgranular zone (SGZ) (Jin and Galvan, 2007; Pino et al., 2017) of the hippocampus. Brain injury, such as ischemic stroke, can activate endogenous NPCs (eNPCs) proliferate and migrate to injury area, and then, to an extent, promote neurogenesis and compensate for neuron necrosis (Zhang and Chopp, 2009; Lin et al., 2015). Unfortunately, this compensatory function is very limited (Apple et al., 2017; Zuo et al., 2019). Thus, activation of endogenous neurogenesis can play an important role in the promotion of neurological function recovery, reflecting great clinical application value.

Reelin is an extracellular glycoprotein that exerts regulating neuronal cell proliferation, migration, and is involved in modulating synaptic function (Folsom and Fatemi, 2013; Wasser and Herz, 2017). Tau is a microtubule-associated protein, which contributes to microtubule aggregation and stability, the development of nerve cells, and the transport of axons (Ebneth et al., 1998; Biernat and Mandelkow, 1999). Abnormal hyperphosphorylation of tau protein has been reported after cerebral ischemia/reperfusion, resulting in microtubule depolymerization and ultimately neuron apoptosis (Ali and Kim, 2015; Zhu et al., 2018). Studies have revealed that tau-deficient mice are protected from neurological deficits and have less infarct volume following experimental ischemic stroke (Bi et al., 2017). Reelin is reported to control tau phosphorylation through ApoE-receptor 2/disabled-1/GSK-3β in neurodegeneration diseases, such as Alzheimer’s disease (Ohkubo et al., 2003), but this neuroprotective effect is still unclear in ischemic stroke.

Traditional Chinese medicine has been used for ischemic stroke for millennia (Li et al., 2016; Seto et al., 2016). Sanhua Decoction (SHD) is a representative traditional Chinese medicine formula for ischemic stroke, which was first collected in *Suwen Bingji Qiyi Baomingji* (1115-1368). The prescription consists of four herbs, *Dahuang* (Radix et Rhizoma Rhei), *Qianghuo* (Rhizoma et Radix Notopterygii), *Houpu* (Cortex Magnoliae Officinalis) and *Zhishi* (Fructus Aurantii Immaturus), in a ratio of 4:2:2:1.5, which is still widely used for stroke in modern times (Yang et al., 2009; Liu, 2011). Our previous studies showed that SHD can effectively improve the NIHSS score and Glasgow score in patients with ischemic stroke (Lu et al., 2014) and reduce infarct volume (Dai et al., 2011), brain water content, as well as improving neurological deficits in animals (Lu et al., 2015). However, whether SHD exerts neuroprotective effect by regulating reelin/tau pathway and promoting eNPCs remains unclear. Thus, in the present study, we aim to investigate the effects of SHD on reelin/tau pathway and promoting endogenous neurogenesis in cerebral ischemia/reperfusion (CIR) injury rat models.

## Materials and Methods

### Ethics Statement

All animals were obtained from the Shanghai Laboratory Animal Center (SCXK, 2010-0002). The protocol was approved by the local ethics committee of the Wenzhou Medical University (wydw2015-0148). Procedures involving animals and their care were conducted in accordance with the National Institutes of Health Guide for the Care and Use of Laboratory Animals (Publication No. 85-23). All the animals were sacrificed by anesthesia at the end of the experiment. The utmost possible efforts were made to reduce the number of animals used and minimize animal suffering.

### Experimental Animals

All adult male Sprague-Dawley (SD) rats (body weight, 250–280 g; age, 7–8 weeks) were randomly divided into three groups: Sham group, CIR group, and SHD group, and each group was further divided into subgroups according to different time points (6 h, 1, 3, 7, 14, 21, and 28 d) after CIR. All animals housed in the polycarbonate cages with temperature of 21–25°C, humidity around 50%, a 12-h alternating light/dark cycle (lights on at 08:00–20:00), free access to food and water, and weighed once daily. All studied subjects were adapted to the investigators for 5 d prior to the experiment.

### Animal Models

CIR injury was performed in SD rats according to the well-recognized method (Longa et al., 1989). In brief, after 12-h fast, SD rats were anesthetized with 10% chloral hydrate (300 mg/kg) though intraperitoneal injection. A midline incision was performed on the neck to expose the right common carotid artery (CCA), external carotid artery (ECA), and internal carotid artery (ICA). After ligation of ECA, a monofilament nylon suture with a diameter of 0.26 mm (Beijing Shadong Bio Technologies Co., Ltd., China) was inserted from the ECA to occlude the MCA until a resistance appeared (depth, 19 ± 0.5 mm). After 2-h occlusion with body temperature preservation by a heating blanket, the monofilament nylon suture was withdrawing to restore the brain blood flow of ischemic area. All rats in Sham group were isolated the right CCA and ICA but no MCA occlusion was performed.

### Drugs and Administration

SHD was prepared according to our previous study (Lu et al., 2015). *Dahuang* (Radix et Rhizoma Rhei), *Qianghuo* (Rhizoma et Radix Notopterygii), *Houpu* (Cortex Magnoliae Officinalis), and *Zhishi* (Fructus Aurantii Immaturus) were purchased from Guangdong Yifang Pharmaceutical Co., Ltd. (Guangzhou, China) and mixed at 4:2:2:1.5 by dry weight. The product of quality control was also carried out by the company. The prescription was prepared equal to dry weight of raw materials into 1 g/ml before use every time. 5-Bromo-2-deoxyuridine (BrdU) was provided by Sigma (B5002) and dissolved in normal saline by 20 mg/ml, storing at 4°C until use.

Intragastrical administration of SHD (10 g kg^–1^ d^−1^ for SHD group) or normal saline (same volume for Sham and CIR groups) was performed once a day beginning at 3 d before the surgery until the rats were sacrificed. In order to test the proliferation of eNPCs, BrdU was injected intraperitoneally at the dose of 50 mg/kg once per 4 h for three times, 24 h before sacrifice. To test the differentiation and migration of eNPCs, BrdU was injected intraperitoneally twice a day for 3 d at the dose of 50 mg/kg after surgery. Flow diagram of the experimental protocols was showed in Figure 1.

**Figure 1:** Flow chart of the experimental protocols.

### Neurological Deficit Scores

Behavior assessment was blindly performed after reperfusion at each time point (6 h, 1, 3, 7, and 14 d) with a five-grade scale (Longa et al., 1989) as follows: 0, no obvious neurological deficits; 1, failure of stretching the contralateral forelimb fully when lifting the rats’ tail; 2, circling toward the unaffected side when crawling forward; 3, leaning toward the unaffected side when crawling forward; 4, no spontaneous locomotion, loss of consciousness, or death. Only rats meeting 1–3 points after 2 h of occlusion were considered successful models and then included in subsequent researches.

### Immunofluorescence Staining

At each time points, rats were deeply anesthetized with 10% chloralhydrate (400 mg/kg), thoroughly perfused with saline and precooled 4% paraformaldehyde. Then, brains were removed quickly, excised cerebellum, brainstem and the front half of the brain, cut coronally, retained brain tissue starting from optic cross, and fixed overnight with paraformaldehyde at 4°C. After washed with water overnight, brain sections were dehydrated with increasing graded ethanol (70, 80, 90, 95, and 100%), cleared twice in xylene for 30 min each, embedded in paraffin, and then cut to 5 μm sections. We reserved one section for every three sections for subsequent staining.

Brain slides were then incubated for 1 h at 60°C, dewaxed twice with xylene for 15 min each, then hydrated with graded ethanol (100, 90, 80, and 70%) and water for 3 min, respectively. Endogenous peroxidase elimination was conducted in 3% H_2_O_2_ for 10 min and then rinsed with PBS. Slides were then treated with 0.01 mol/L citrate buffer for 5 min under high temperature and pressure before rinsed with PBS. After antigen retrieval, slides were incubated in 2 mol/L HCL for 20 min at 37°C, followed by 0.1 mol/L sodium borate solution for 10 min at room temperature, before rinsed with PBS. Blocking the slides with 10% Donkey serum for 1 h at room temperature, then sheep anti-BrdU (1:300, ab1893, Abcam), rabbit anti-DCX (1:800, ab18723, Abcam), and rabbit anti-GFAP (1:1,000, ab7260, Abcam) were used to incubate slides at 4°C overnights. After rinsing with PBS, slides were incubated with secondary antibodies for 1 h at 37°C. Covering with anti-fade mounting medium and coverslips, slides were then examined by a fluorescence microscope. There were six rats in each group, and five discontinuous sections of each rat were finally included. The number of positive cells was counted by Image-pro Plus 6.0, and the mean value was used as the result at each time point.

### Western Blot

Affected hippocampal tissues were lysed in ice-cold RIPA buffer (Beyotime, China), containing PMSF (Beyotime, China) and phosphatase inhibitor (Solarbio, China). Total protein concentration was determined by the BCA protein assay (Beyotime, China). Aliquots of homogenate with equal protein concentration were separated by 10% SDS-PAGE gel and then transferred to polyvinyl difluoramine membrane. After blocking in 5% non-fat milk for 1.5 h at room temperature, the membranes were then incubated with primary antibodies, including mouse anti-reelin (1:1,000, ab78540, abcam), mouse anti-tau (tau-5, 1:5,000, ab80579, abcam), and rabbit anti-tau (phospho-S199/202, 1:5,000, ab4864, abcam) at 4°C overnight. The blots were then incubated with anti-rabbit or anti-mouse IgG conjugated to HRP for 2 h at room temperature and visualized using the enhanced chemiluminescence.

### Real-Time Quantitative Reverse Transcription Polymerase Chain Reaction

Total RNA was isolated from affected hippocampal tissues using Trizol reagent (Invitrogen) before being reverse transcribed into cDNA using Prime Script TM RT reagent Kit (TAKARA). Then RT-qPCR was performed using SYBR R Premix Ex TaqTMII (TAKARA) and gene-specific primers on a Light Cycler thermal cycler system (Bio-Rad). The gene-specific primers were as follows: reelin: forward, 5′-TGGGATAACATGGAAACTCTTGGAG-3′ and revised, 5′-ACCATCTGAACTGGATTCCAAACTG-3; tau: forward, 5′-CCAGGAGTTTGACACAATGGAAGAC-3′ and revised, 5′-CTGCTTCTTCAGCTTTTAAGCCATG-3′; GAPDH: forward, 5′-ATCGCCAGTCCGTCTTCTACATC-3′ and revised, 5’-TGATCGTGGTGACTCCCATCC-3′.

### Statistical Analysis

Graph Pad Prism (Graph Pad, USA) was used for statistical analyses and results were expressed as means ± standard deviation (mean ± SD). One-way analysis of variance (ANOVA) was used to analyze differences between multiple groups and *t*-test was used to analyze differences between two groups. Significant difference was considered when *p* < 0.05.

## Results

### Effect of Sanhua Decoction on Neurological Deficits

There was no sign of neurological deficits in Sham group (scored 0 points at each time point). Compared with Sham group, CIR group had an increased NDS at each time point (*p* < 0.05), which peaked at 3 d. Compared with CIR group, SHD group had a significant decrease on NDS at 1, 3, 7, and 14 d (*p* < 0.05), despite that at 6 h (*p* > 0.05) (Figure 2).

**Figure 2:** The neurological deficit scores in the Sham, CIR, and the SHD group at 6 h, 1, 3, 7, and 14 d after reperfusion in rats (*n* = 6). ^*^p < 0.05, compared to the Sham group; ^#^*p* < 0.05, compared to the CIR group.

### Effect of Sanhua Decoction on the Number of BrdU Positive Cells in Subventricular Zone

There was no significant difference on the number of BrdU positive cells in SVZ in Sham group at each time point. In both CIR and SHD groups, the number of BrdU positive cells in SVZ reached a peak at 7 d after reperfusion (Figures 3B,E). Compared with Sham group, the number of BrdU positive cells showed a significant increase in CIR group at 3, 7, and 14 d (*p* < 0.01) (Figures 3A–C,E) and in SHD group at 3, 7, 14, and 21 d (*p* < 0.01) (Figures 3A–E). Compared with CIR group, SHD showed a significant increase on the number of BrdU positive cells at 3, 7, and 14 d (*p* < 0.05) (Figures 3A–C,E). There was no difference comparing CIR group with Sham or SHD group at 21 d (*p* > 0.05).

**Figure 3:** Immunofluorescence staining of BrdU positive and BrdU/DCX positive cells in the subventricular zone (SVZ) of the Sham, CIR and SHD groups at 3 d **(A)**, 7 d **(B)**, 14 d **(C)**, and 21 d **(D)** after reperfusion (*n* = 6; scale bar = 100 μm). **(E)** The bar graph of the number of BrdU positive cells. **(F)** The bar graph of the number of BrdU/DCX positive cells. ^*^p < 0.05, ^**^p < 0.01, compared to the Sham group; ^#^*p* < 0.05, ^##^*p* < 0.01, compared to the CIR group.

### Effect of Sanhua Decoction on the Number of BrdU/DCX Positive Cells in Subventricular Zone

There was no significant difference on the number of BrdU/DCX positive cells in SVZ in Sham group at each time point. The number of BrdU/DCX positive cells in SVZ reached a peak at 7 d in both CIR and SHD groups (Figures 3B,F). Compared with Sham group, BrdU/DCX positive cells showed a significant increase in CIR group at 7 and 14 d (*p* < 0.05) (Figures 3B,C,F) and in SHD group at 3, 7, and 14 d (*p* < 0.01) (Figures 3A–C,F). Compared with CIR group, the number of BrdU/DCX positive cells had a significant increase in SHD group at 3, 7, and 14 d (*p* < 0.05) (Figures 3A–C,F). However, there was no significant difference between three groups at 21 d after reperfusion (*p* > 0.05).

### Effect of Sanhua Decoction on the Number of BrdU/GFAP Positive Cells in Ischemic Penumbra

The number of BrdU/GFAP positive cells in ischemic penumbra showed an upward trend. Compared with CIR group, there was a significant difference in SHD group at 28 d after reperfusion (*p* < 0.01) but with no difference at 14 d (*p* > 0.05) (Figure 4).

**Figure 4:** Immunofluorescence staining of BrdU/GFAP positive cells in the ischemic penumbra of the CIR and SHD groups at 14 d **(A)** and 28 d **(B)** after reperfusion (*n* = 6; scale bar = 100 μm). **(C)** The bar graph of the number of BrdU/GFAP positive cells. ^##^*p* < 0.01, compared to the CIR group.

### Effect of Sanhua Decoction on the Expression of Reelin, Total Tau, and Phosphorylated Tau

We evaluated the expression of reelin, total tau (t-tau), and phosphorylated tau (p-tau) by western blot and RT-qPCR. The present results showed that the protein and mRNA levels of reelin (Figure 5) and t-tau (Figure 6) had no significant differences comparing SHD group with Sham or CIR groups among all the time point. In terms of the expression of p-tau (Figure 7), there was a significant increase in CIR group among the time point of 6 h, 1, 3, 7, and 14 d comparing with that of Sham group (*p* < 0.05). In SHD group, p-tau significantly decreased at 1, 3, 7, and 14 d after reperfusion when compared with that of CIR group (*p* < 0.05).

**Figure 5:** The expression of reelin in hippocamp in the Sham, CIR and the SHD group at 6 h, 1d, 3d, 7d and 14d after reperfusion in rats (*n* = 6). **(A)** The results from the western blot. **(B)** Quantitative analysis for the protein level of reelin. **(C)** Quantitative analysis for the mRNA level of reelin.

**Figure 6:** The expression of total tau in hippocamp in the Sham, CIR, and the SHD group at 6 h, 1d, 3d, 7d and 14d after reperfusion in rats (*n* = 6). **(A)** The results from the western blot. **(B)** Quantitative analysis for the protein level of t-tau. **(C)** Quantitative analysis for the mRNA level of t-tau.

**Figure 7:** The expression of phosphorylated tau in hippocamp in the Sham, CIR and the SHD group at 6 h, 1d, 3d, 7d and 14d after reperfusion in rats (*n* = 6). **(A)** The results from the western blot. **(B)** Quantitative analysis for the protein level of p-tau. ^*^p < 0.05, compared to the Sham group; ^#^*p* < 0.05, compared to the CIR group.

## Discussion

The main findings of this study suggested that SHD can significantly improve neurological deficit, decline p-tau expression, and increase the number of BrdU positive and BrdU/DCX positive cells in SVZ and the number of BrdU/GFAP positive cells in the ischemic penumbra. SHD exerted neuroprotective effects through downregulating of p-tau and promoting neurogenesis by eNPCs’ proliferation, migration, and differentiation.

Neuronal necrosis is hardly to avoid in acute brain injury such as ischemic stroke (Zuo et al., 2019). Due to there is lack of neuroprotective drug can reverse neurological deficits for now, cell-based therapies, which substantially enhance neurobehavioral recovery, is widely concerned (Bernstock et al., 2017; Boese et al., 2018). Preclinical studies have demonstrated that exogenous stem cells transplantation can not only promote the recovery of motor function but also improve the cognitive function in CIR models (Chen et al., 2014; Wei et al., 2017). However, there are still some faultiness, like unstable cell source, uncertain differentiation endpoint, and lack of long-term evidence (Wislet-Gendebien et al., 2012). Endogenous NPCs can be activated by ischemic brain injury, then proliferate, differentiate, migrate, and finally replace the necrotic neurons, restoring neurological function effectively (Nakatomi et al., 2002; Sun et al., 2004). Thus, mobilizing eNPCs can be a new approach to the treatment of cerebral ischemic stroke. In the present study, we found the number of BrdU positive cells in SVZ increased within the first week but declined during the next 2 weeks, which is in accordance with previous studies (Zhang et al., 2001; Kernie and Parent, 2010). SHD can further upregulate new born cells at each time points after CIR. We also found the number of BrdU/DCX positive cells in SVZ showed a similar trend compared to BrdU positive cells, reaching a peak at 7 d after CIR. SHD promoted this change, suggesting that it can facilitate eNPCs differentiate into immature neurons.

Brain injury can activate eNPCs and promote their migration from the SVZ into the injured region. Studies have revealed the related factors such as stromal cell-derived factor 1 (SDF-1) and CXC chemokine receptor 4 (CXCR4) (Parent et al., 2002; Ohab et al., 2006) and monocyte chemoattractant protein-1 (MCP-1) and CC chemokine receptor 2 (CCR2) (Yan et al., 2007). After ischemic stroke, SDF-1α increases highly and reaches a peak at 7–14 d after ischemia, which promotes the directional movement of neural progenitors to the injured area for neurogenesis (Stumm et al., 2002; Ohab et al., 2006; Robin et al., 2006). At the meantime, the administration of SDF-1 receptor CXCR4 antagonists suppresses the migration (Parent et al., 2002), causing neuroblasts to spread non-directionally to the cortex (Ohab et al., 2006). It has also been reported that MCP-1/CCR2 signaling promotes the directed migration of NPCs toward the infarct region both *in vitro* (Liu et al., 2007) and transplantation (Yan et al., 2007) studies. Microglia, oligodendrocytes, and astrocytes are three main types of glia in the CNS, while the number of astrocytes is the highest, accounting for about 20–50% (Lanciotti et al., 2013). Recently, it has been found that astrocytes play multiple roles in the physiological functions of brain. Astrocytes maintain a stable environment within the CNS by regulating the concentrations of ions, water, neurotransmitters, neurohormones, energy, and metabolites (Belanger et al., 2011). Astrocytes are also involved in neural regeneration, synapse generation, and the formation and maintenance of the blood-brain barrier (Abbott et al., 2006; Perea et al., 2009; Lanciotti et al., 2013). Studies have found that there is a close relationship between astrocytes and neurons (Logica et al., 2016; Rose and Chatton, 2016). The migration, survival, and formation of synaptic connections in neonatal neurons require the guidance and support of astrocytes. Studies have shown that astrocytes proliferate actively after cerebral ischemia that can fill brain tissue defects after neuron damage, engulf necrotic tissue fragments, provide energy to neurons, and secrete a variety of neurotrophic nutrients (Pekny et al., 2016). It can also reduce the toxic effects of some molecules, such as glutamic acid, on neurons to protect the injured neurons (Mahmoud et al., 2019). GFAP is an astrocyte-specific antigen marker, in this study, we found that SHD significantly increased ischemic penumbra BrdU/GFAP positive cells at 28 d after CIR, suggesting that SHD can promote the differentiation of eNPCs into astrocytes and facilitate their migration.

Tau contributes to stabilize the structure of microtubules, maintaining the morphology of neurons (Avila et al., 2004). The accumulation of soluble hyperphosphorylated tau forms neurofibrillary tangles, disrupting the ability of binding microtubules and promoting aberrant tau aggregation, which may underlie tau-mediated neurodegeneration (Min et al., 2010). Cerebral ischemia/reperfusion can induce tau hyperphosphorylation, resulting in decreased microtubule stability, reduced neuronal activity and eventually cell death (Basurto-Islas et al., 2018). Moreover, stabilization of microtubule and cytoskeleton plays an important role in eNPCs proliferation, migration, and differentiation (Jaglin and Chelly, 2009). Therefore, suppression of aberrantly phosphorylated tau can be a therapeutic approach for ischemic stroke. In this study, we found that SHD could significantly reduce p-tau level at 1, 3, 7, and 14 d after reperfusion compared with CIR group, while there was no significant change on t-tau protein and mRNA levels, suggesting that SHD exerts neuroprotective and promoting neurogenesis effects *via* reducing tau phosphorylation.

Reelin is an extracellular matrix protein synthesized by Cajal-Retzius cells. Reelin signaling is reported to regulate microtubule dynamics by binding to ApoER2 receptors and inhibiting GSK-3β activity, which is known to be an important phosphatase of tau (Chai and Frotscher, 2016). In our study, there was no difference on reelin protein and mRNA levels at each time point after reperfusion between Sham group and CIR group, which is in accordance with the recent study (Lane-Donovan et al., 2016). SHD also had no effect on the expression level of reelin in CIR, illustrating that SHD may regulate p-tau level though the downstream molecules of reelin signaling. Further research is needed to explore the specific mechanisms of SHD on controlling tau pathological state in different stages of stroke.

In the present study, we used SD rats aged 7–8 weeks. Although ischemic stroke is more likely to occur in the elderly in clinic, many studies currently published in high-impact factor journals, such as Stroke and Journal of Cerebral Blood Flow and Metabolism, are still based on young rats (Suh et al., 2015; Liu da et al., 2016; Khodanovich et al., 2018; Qin et al., 2019) for the following reasons: the overall mortality rate of elderly rats after 60-min middle cerebral artery occlusion (43.5%) is significantly higher than that of the young rats (6.3%); there is no meaningful difference in the infarct volume between the young and old rats at 24 h or 28 d after ischemia, suggesting that comparing with a young rat, the recovery would be of no difference if an old rat survives in a short period after the MCAO procedure (Wang et al., 2003). Thus, we used young SD rats in the present study. We will try to include elderly animals to get closer to the clinical status of ischemic stroke in the future.

In this study, we mainly investigated the effect of SHD on promoting the proliferation and migration, and the differentiation into glia of eNPCs in CIR injury, without further research into the differentiation into mature neurons, which is the limitation in this study as well as our future research directions.

## Conclusion

The present study indicates that SHD can improve NDS and promote neurogenesis by eNPCs’ proliferation, migration, and differentiation. SHD exerts neuroprotective effects against cerebral ischemia/reperfusion injury through downregulation of p-tau, which may help to the future development of therapeutic strategies.

## Data Availability Statement

All datasets generated for this study are included in the article/supplementary material.

## Ethics Statement

The animal study was reviewed and approved by the ethics committee of the Wenzhou Medical University.

## Author Contributions

D-LF, J-HL, Y-HS, YL, and G-QZ contributed in study conception and design. D-LF, J-HL, Y-HS, and X-LZ conducted experiments and helped in data analysis and/or interpretation. D-LF, J-HL, and Y-HS supervised the study and wrote the manuscript. All authors participated in the final approval of the version to be published.

### Conflict of Interest

The authors declare that the research was conducted in the absence of any commercial or financial relationships that could be construed as a potential conflict of interest.

## Abbreviations

BrdU: 5-Bromo-2-deoxyuridine
CCA: Common carotid artery
CCR2: CC chemokine receptor 2
CIR: Cerebral ischemia/reperfusion
CNS: Central nervous system
CXCR4: CXC chemokine receptor 4
d: Days
ECA: External carotid artery
eNPCs: Endogenous neural precursor cells
h: Hours
ICA: Internal carotid artery
MCP-1: Monocyte chemoattractant protein-1
min: Minutes
NDS: Neurological deficit scores
NPCs: Neural precursor cells
NS: Normal saline
NSCs: Neural stem cells
SD: Sprague-Dawley
SDF-1: Stromal cell-derived factor 1
SGZ: Subgranular zone
SHD: Sanhua Decoction
SVZ: Subventricular zone
